The article "Artificial Intelligence-Based Approach for Misogyny and Sarcasm Detection from Arabic Texts" was published in 2022. Journal: Comput Intell Neurosci.

# Artificial Intelligence-Based Approach for Misogyny and Sarcasm Detection from Arabic Texts

**DOI:** 10.1155/2022/7937667

**Published:** 2022-03-26

**Authors:** Abdullah Y. Muaad, Hanumanthappa Jayappa Davanagere, J. V. Bibal Benifa, Amerah Alabrah, Mufeed Ahmed Naji Saif, D. Pushpa, Mugahed A. Al-antari, Taha M. Alfakih

**Affiliations:** ^1^Department of Studies in Computer Science, University of Mysore, Manasagangothri, Mysore 570006, India; ^2^Sana'a Community College, Sana'a 5695, Yemen; ^3^Department of Computer Science and Engineering, Indian Institute of Information Technology, Kottayam, India; ^4^Department of Information Systems, College of Computer and Information Sciences, King Saud University, Riyadh 11543, Saudi Arabia; ^5^Department of Computer Applications, Sri Jayachamarajendra College of Engineering (Affiliated to VTU University), Mysore, India; ^6^Department of Information Science and Engineering, Maharaja Institute of Technology Mysore, Mysore, Karnataka, India; ^7^Department of Artificial Intelligence, Daeyang AI Center, Sejong University, Seoul 05006, Republic of Korea; ^8^Faculty of Engineering and Information Technically, Aljanad University for Science and Technology, Taiz, Yemen

## Abstract

Social media networking is a prominent topic in real life, particularly at the current moment. The impact of comments has been investigated in several studies. Twitter, Facebook, and Instagram are just a few of the social media networks that are used to broadcast different news worldwide. In this paper, a comprehensive AI-based study is presented to automatically detect the Arabic text misogyny and sarcasm in binary and multiclass scenarios. The key of the proposed AI approach is to distinguish various topics of misogyny and sarcasm from Arabic tweets in social media networks. A comprehensive study is achieved for detecting both misogyny and sarcasm via adopting seven state-of-the-art NLP classifiers: ARABERT, PAC, LRC, RFC, LSVC, DTC, and KNNC. To fine tune, validate, and evaluate all of these techniques, two Arabic tweets datasets (i.e., misogyny and Abu Farah datasets) are used. For the experimental study, two scenarios are proposed for each case study (misogyny or sarcasm): binary and multiclass problems. For misogyny detection, the best accuracy is achieved using the AraBERT classifier with 91.0% for binary classification scenario and 89.0% for the multiclass scenario. For sarcasm detection, the best accuracy is achieved using the AraBERT as well with 88% for binary classification scenario and 77.0% for the multiclass scenario. The proposed method appears to be effective in detecting misogyny and sarcasm in social media platforms with suggesting AraBERT as a superior state-of-the-art deep learning classifier.

## 1. Introduction

Posts and tweets on social media platforms allow people to share their thoughts, emotions, and sentiments. Regularly, Internet bullying is observed, which is considered a form of attacking, and it has escalated against people [1, 2]. with a growth in the number of people using social media sites such as Twitter to express themselves [3]. The lack of tools and benchmark datasets are the main challenges in this field [4]. The goal here is to construct an accurate method for detecting misogyny and sarcasm from Arabic text. The limitation of studies in Arabic context serves as motivation to research and build practical smart solutions through the design and development of automatic identification systems [5].

There are around 447 million native speakers who speak Arabic as their first language, with many more speaking it as a second or religious language. As a result, Arabic has become one of the world's most frequently spoken languages. At the same time, Arabic is the primary language of 22 Arab countries and many other Islamic countries. The writing of Arabic is written from right to left. It is the world's fifth most spoken language [6–8]. Arabic has a rich morphology and a complex orthography [9].

Text detection is one of the big challenges of NLP which still has many limitations to work with, especially for the Arabic language when compared to English. There are many types of text detection such as prediction of human behavior [10], hate speech detection [11], exploring halal tourism [12], gender detection [13], misogyny detection [14], sarcasm detection [15], detection and classification of psychopathic personality [16], fake news detection [17], and detection of dialectal in the Arabic language [18]. This study aims to design a model for automatically detecting misogyny and sarcasm using machine learning (ML) and deep learning (DL) methods with different benchmark datasets [19, 20].

The proposed study is evaluating state-of-the-art deep learning classifiers for multiple topics (i.e., misogyny and sarcasm) at the same time. Whereas most Arabic text detection latest studies were focusing only on a single topic. The requirements to develop a method for detecting any type of Arabic text, such as sarcasm and hate speech, represent the Arab society needs. It is critical since our system must be able to reliably detect any suspicious text. The contributions for this work are summarized as follows:

- A comprehensive study is performed via seven ML/DL classifiers with two scenarios: binary and multiclass classification problems
- Two different datasets are used to evaluate the proposed research concept for distinguishing Arabic misogyny and sarcasm from Arabic tweets
- Multiple topics of misogyny and sarcasm are simultaneously detected via the proposed scenarios
- The proposed study investigates the best deep learning classifier for Arabic texts in terms of increasing the surfing life on social media networks

The remainder of this paper is organized as follows: In Section 2, we address the related works in misogyny and sarcasm identification in Arabic.  Section 3 illustrates the suggested model and model architecture. Following that, in Section 4, we present the experimental analysis. After that, the discussion will be given in Section 5, and the conclusion will be presented with a brief summarization about the future work in Section 6.

## 2. Related Works

Detecting sarcasm text is one of several tasks in NLP. There exist some work in the literature, which has been done for Arabic text detection. As we mention above, there are many types of sarcasm detection of Arabic text, and where we plan to survey some of these works is as follows:

Detection of Arabic text is still in its early stages [21]. Lichouri et al. in [22] presented a comparison between two LSVC and BiLSTM classifiers for Arabic text detection. They presented an intuitive but straightforward detection system based on different stages and combinations. Mulki and Ghanem in [2] introduced an Arabic Levantine Twitter dataset for Misogynistic language (LeT-Mi) to be the first benchmark dataset for Arabic misogyny. Muaad et al. in [23] presented a model to detect misogyny from Arabic text and compare between machine and deep learning algorithms. Al-Yahya et al.in [24] made a comparative study of representation transformer-based language and classification neural network models to detect text in general. Gaanoun and Benelallam in [25] designed a new system using a hybrid ensemble of Gaussian Naive Bayes, MarBERT, and Mazajak embedding. This study has got an F1-sarcastic score of 51% on sarcasm and an F1-PN of 71% for sentiment detection. Husain and Uzuner in [26] designed the system to detect sarcasm and sentiment analysis for Arabic text. Naski et al. in [27] designed a system to classify sentiment for four languages and to detect sarcasm using (mBERT, AraBERT, ARBERT, and MARBERT). Talafha et al. in [28] tried to solve the problem of sarcasm detection from Arabic texts using different methods. The work solves the task as a regression problem; also, this paper finds sarcasm in a given tweet. Faraj et al. in [29] joined the shared task on sarcasm and sentiment detection for the Arabic language. Their goal was to detect whether a tweet was sarcastic or not. They have used an AraBERT pretrained model with an ensemble technique. Their model achieved an accuracy score of 0.78, 30 in this competition. Abuzayed and Al-Khalifa in [30] implemented seven DL models by using an augmentation technique. Their models were able to detect whether a tweet is a sarcasm or not. Wadhawan in [31] used the ArSarcasm-v2 dataset. They processed it by altering different parts of the text. Then, experiments with AraELECTRA and AraBERT transformer-based models have been conducted. The tasks of sarcasm and sentiment detection have been conducted. Abu Farha et al. in [32] provided an overview of the new ArSarcasm-v2 dataset, which is used for the shared task. They also provided a high-level description of the top participating teams in the shared task. In the end, the best 0.62 F1-score and 0.74 FPN results for both sarcasm detection and sentiment analysis tasks have been registered. El Mahdaouy et al. in [33] introduced an end-to-end deep MTL model, allowing knowledge interaction between the two tasks. According to our relevant research, there are limited studies in detecting Arabic text for more than one topic simultaneously, and detection text can contain many topics.

## 3. Proposed Model

### 3.1. Architecture of the Proposed Deep Learning Framework for Arabic Texts

The architecture stages of the misogyny and sarcasm detection approach are given in Figure 1. It consists of three main steps: dataset preparation and splitting, Arabic text representation, misogyny and sarcasm detection, and evaluation scenarios.

The preparation text for further processing can be performed through the preprocessing step. Then, Arabic word representation and feature extraction steps could be performed. Finally, the classification part is performed for both binary and multiclass scenarios.

### 3.2. Preprocessing

Text must be preprocessed in order to be more useful for representation and learning tasks. Preprocessing is a technique for converting data into a specified input data format that might be useful for ML and DL techniques. The primary goal of preprocessing is to remove punctuation, slang, stop words, and other unwanted words that exist in text data. The identification performance of the Arabic misogyny and sarcasm detection task may be harmed by this unpleasant word in the Arabic language. Through a preprocessing phase, we exclude any non-Arabic terms, stop words, and punctuations in this work. Most of the time, we need to work with different preprocessing or combinations of them as we have performed here by using tokenization and stemming. A good text representation can be learned using a variety of conventional and advanced preprocessing approaches [34, 35]. Tokenization is the process of dividing a text into words, phrases, or characters called tokens. Whereas here, the model converts a text (sentence) into words. Then, these words will be converted to weights or embedding vectors depending on which representation we will select. Then, stop word removal has been performed with machine learning.

### 3.3. Arabic Text Representation (Feature Extraction)

Preprocessing data will be ready for representation purposes. Various feature extraction models are used in this section. In the experimental part, the performance was poor with BoW for a machine learning method due to the loss of semantic and syntactic information between words. As a result, we use another representation technique known as AraBERT to handle semantics and syntactic which increase performance by increasing accuracy. The BoW is merely a one-hot encoding extension. It is utilized in a variety of fields, such as NLP. The semantic relationship between words, as well as the order of words and grammar, is neglected in the matrix of words created with BoW. We will explore the other type of representation in the next section.

### 3.4. Arabic Text Classification

Text is recognized and classified to a right label called a classification task. Several algorithms have been implemented here, as we will discuss in Section 5. We will explore different ML and DL techniques called AraBERT. BERT refers to bidirectional encoder representations from transformers which is a contextualized word representation employed in various domains, including natural language understanding, sentiment analysis, and natural language generation, such as text translation. The BERT training is based on two tasks. The first task is a masked language model, and the second task is the next sentence prediction. We adopted the AraBERT model proposed in [36], which is an effective model for the Arabic language text representation and classification task. We implemented some classifiers such as passive-aggressive classifier as (PAC), logistic regression classifier (LRC), random forest classifier (RFC), linear SVC classifier (LSVC), decision tree classifier (DTC), and K nearest neighbor classifier (KNNC).

## 4. Experimental Analysis

### 4.1. Dataset

To evaluate the proposed AraBERT and different ML for detecting misogyny and sarcasm, two Arabic datasets are simultaneously used. Both datasets are prepared for binary and multiclass problems for each topic (i.e., sarcasm or misogyny detection problem). Both datasets are split for training validation with 70% and testing with 30%. The dataset details are demonstrated in the following sections.

#### 4.1.1. Misogyny Dataset

The misogyny dataset is prepared for binary and multiclass problems, as shown in Tables 1 and 2.  Table 1 shows the misogyny data distribution in the case of binary classification scenarios (i.e., non-misogyny vs. misogyny).

Whereas, Table 2 shows the misogyny data distribution in case of multiclassification problem. In this case, eight different classes are considered which are discredit, stereo typing and objectification, damning, threat of violence, derailing, dominance, sexual harassment, and non-misogyny.

#### 4.1.2. Sarcasm Dataset

In the same way, the sarcasm dataset is prepared for binary and multiclass problems. Tables 3 and 4 show the detail of data distribution per class for the binary and multiclass scenarios, respectively.

### 4.2. Implementation Environment

The experiments of this study are performed using deep learning Google Collab environment with different libraries such as NLTK, pandas, sci-kit-learn (https://scikit-learn.org/stable/), TensorFlow (https://www.tensorflow.org/), transformer (https://huggingface.co/docs/transformers/index), and Keras (https://keras.io/). Several ML and DL models are adopted and implemented to achieve the goal of this study such as AraBERTv2, ARABERT, PAC, LRC, RFC, LSVC, DTC, and KNNC. These algorithms are deployed for both misogyny and sarcasm detection from Arabic tweets on social networks. The datasets (https://github.com/bilalghanem/let-mi) and codes are available on GitHub (https://github.com/abdullahmuaad8).

### 4.3. Evaluation Metrics

For this study, the evaluation metrics of recall, precision, *F*1-score, and accuracy are used. The mathematical definition of these indices are expressed as follows:

(1) $$\begin{array}{c} \text{Recall}=\;\frac{\text{TP}}{\text{TP}+\text{FN}},\\ \mathrm{Pr}\text{ecision}=\;\frac{\text{TN}}{\text{TN}+\text{FP}},\\ F1-\text{score }=\;\frac{2\text{TP}}{2\text{TP}+\text{FP}+\text{FN}},\\ \text{Accuracy }=\;\frac{\text{TP}+\text{TN}}{\text{TP}+\text{FN}+\text{TN}+\text{FP}}\;. \end{array}$$

where TP refers to true positives, TN refers to true negatives, FP refers to false positives, and FN refers to false negatives. These parameters are derived using the confusion matrices for both classification scenarios: binary and multiclass problems [36–40].

## 5. Discussion and Results

This part highlights that the results and discussions of the different methods have been used describing the several trials with two different datasets. These experimentations are focused on two tasks: binary classification and multiclassification for both misogyny and sarcasm.

### 5.1. Misogyny Detection

#### 5.1.1. Misogyny Binary Classification

Table 5 and Figure 2 show the results of the misogyny detection for binary classification. The linear SVC model was better than other ML in terms of accuracy, precision, recall, and *F*-1 score. At the same time, we executed AraBERTv2, as transfer learning algorithm that provides high accuracy but it costs in terms of execution time more than other ML techniques.

#### 5.1.2. Misogyny Multiclass Classification

Multiclassification is more complicated than binary classification, so learning the pattern here is less accurate as we have seen in Table 6. The results of multiclassification have been presented in Table 6 and Figure 3. The linear SVC model performs better than the others in terms of accuracy and the random forest model performs poorly, according to the findings.

Simultaneously, we were using ARABERTv2 that provided outstanding accuracy but required more time than others. Lastly, we do want to point out that an imbalanced dataset will have an impact on categorization accuracy. As we have seen in Table 2, the class dominance contains only 38 comments document after dividing data to train and test the number of documents will be very less and learning about this class will be very less too. So, augmentation of data is recommended for future work.

### 5.2. Sarcasm Detection

#### 5.2.1. Sarcasm Binary Classification

Table 7 and Figure 4 illustrate the results of the sarcasm classification for the sarcasm dataset. The linear SVC model exceeds all ML model in terms of accuracy, precision, recall, and *F*1-score. At the same time, we employed ARABERTv2, that provided good accuracy but took a long time compared to the ML model.

#### 5.2.2. Sarcasm Multiclass Classification

Table 8 and Figure 5 show the outcomes of the multidetection and categorization process. The linear SVC model in terms of *F*1-score outperforms the others, but the logistic regression model in terms of precision was better, and both of the models were equal in terms of accuracy and recall. According to the findings, the performance of the random forest classifier model is weak. At the same time, we used ARABERTv2, that provided great accuracy but consumed more time than the ML approach.

Finally, we would like to draw attention to the fact that the dataset was skewed. For example, as seen in Table 4, the positive class contains only two thousand five hundred, but other classes have more than six thousand, so the learning for these classes will not be same, and working with augmentation technique will be better for getting good accuracy as future work.

From the results in Tables 5 and 6 for the binary classification as well as Tables 5 and 6 for the multiclassification, we see that the accuracy 90% and 89% for binary classification were better than multiclassification which were 82% and 77%, respectively. Finally working with deep learning gives better results but a lack of data and unbalance of the dataset is one of the challenges for researchers in Arabic natural language processing.

## 6. Conclusion

The problem of the sarcasm detection of Arabic text has become a major problem for Arab people. In this work, we introduce a model to detect misogyny and sarcasm from Arabic text. We have carried out our work utilizing two datasets called (misogyny and Abu Farah datasets). Our results provide excellent accuracy equal to 91% and 88% for binary classification, respectively and 82% and 77% for multiclassification, respectively, using the AraBERT deep learning classifier. This work indicates that there are various outstanding issues, starting with finding benchmark datasets and lexicons for Arabic text detection topics. At the same time, data augmentation techniques can be used to address dataset imbalances. Finally, future studies should examine the model to find the relation between various topics and the mixed language problem.

## Figures and Tables

**Figure 1:** Architecture of misogyny and sarcasm detection model.

**Figure 2:** Comparison evaluation results for misogyny binary classification scenario in terms of overall accuracy.

**Figure 3:** Comparison evaluation results for misogyny multiclass classification scenario in terms of overall accuracy.

**Figure 4:** Comparison evaluation results for sarcasm binary classification scenario in terms of overall accuracy.

**Figure 5:** Comparison evaluation results for sarcasm multiclass classification scenario in terms of overall accuracy.

**Table 1:** Misogyny data distribution for binary class scenario

**#**	**Category**	**نوع الصنف**	**No. of Arabic Documents**	**Training**	**Testing**
1.	Non-misogyny	لا توجد كراهية	3,061	2,143	918
2.	Misogyny	كراهية النساء توجد	4,805	3,364	1,442

**Table 2:** Misogyny data distribution for multi-class scenario

**#**	**Category**	**نوع الصنف**	**No. of Arabic Documents**	**Training**	**Testing**
1.	Discredit	تشويه السمعة	2,327	1,629	489
2.	Stereo typing & objectification	الكتابة والصياغة المجسمة	290	203	61
3.	Damning	اللعنة	256	179	54
4.	Threat of violence	التهديد بالعنف	175	123	37
5.	Derailing	الخروج عن السكة	59	41	12
6.	Dominance	هيمنة	38	27	8
7.	Sexual harassment	التحرش الجنسي	17	12	4
8.	Non-misogyny	لا توجد كراهية	3,388	2,372	711

**Table 3:** Sarcasm data distribution for binary class scenario

**#**	**Category**	**نوع الصنف**	**No. of Arabic Documents**	**Training**	**Testing**
1.	Non-sarcastic	لا توجد سخرية	12,559	8,791	3,768
2.	Sarcastic	سخرية	2,989	2,092	897

**Table 4:** Sarcasm data distribution for multi-class scenario

**#**	**Category**	**نوع الصنف**	**No. of Arabic Documents**	**Training**	**Testing**
1.	Positive	سخرية إيجابية	2,577	1,804	773
2.	Negative	سخرية سلبية	6,298	4,409	1,889
3.	Neutral	سخرية معتدلة	6,495	4,547	1,948

**Table 5:** Arabic misogyny detection evaluation results for binary classification task.

Classifier model	Accuracy (%)	Precision (%)	Recall (%)	*F*1-score (%)
PAC	81	84	86	85
LRC	81	81	90	86
RFC	62	62	67	76
LSVC	83	85	88	86
DTC	70	74	78	76
KNNC	65	64	98	78
AraBERT	**91**	—	—	**90**

The bold values represent the highest values of evaluation metrics achieved by the corresponding classifier model.

**Table 6:** Arabic misogyny detection evaluation results for multiclass classification task.

Classifier model	Accuracy (%)	Precision (%)	Recall (%)	*F*1-score (%)
PAC	72	72	72	72
LRC	69	68	68	68
RFC	40	39	39	39
LSVC	74	73	73	**73**
DTC	56	56	56	56
KNNC	44	43	43	43
ARABERT	**82**	—	—	—

The bold values represent the highest values of evaluation metrics achieved by the corresponding classifier model.

**Table 7:** Arabic sarcasm detection evaluation results for sentiment classification task: binary scenario.

Classifier model	Accuracy (%)	Precision (%)	Recall (%)	*F*1-score (%)
PAC	83	81	83	**81**
LRC	83	81	83	77
RFC	82	68	82	74
LSVC	84	82	84	**81**
DTC	78	76	78	77
KNNC	83	79	83	76
ARABERT	**88**	—	—	77

The bold values represent the highest values of evaluation metrics achieved by the corresponding classifier model.

**Table 8:** Detection evaluation results of Arabic sentiment compared with different classifiers: multiclass scenario.

Classifier model	Accuracy (%)	Precision (%)	Recall (%)	*F*1-score (%)
PAC	71	68	71	69
LRC	73	73	73	68
RFC	68	46	66	55
LSVC	73	69	73	70
DTC	63	62	63	63
KNNC	68	59	68	57
ARABERT	**77**	—	—	**75**

The bold values represent the highest values of evaluation metrics achieved by the corresponding classifier model.

## Data Availability

The data used to support the findings of this study are available from the corresponding author upon request.
